The article "Artificial Intelligence Assists the Construction of Quantitative Model for the High-Quality Development of Modern Enterprises" was retracted in 2022. Reason: concerns about the peer review.

# Artificial Intelligence Assists the Construction of Quantitative Model for the High-Quality Development of Modern Enterprises

**DOI:** 10.1155/2021/7211790

**Published:** 2021-11-25

**Authors:** Min Li, Zamira Madina

**Affiliations:** ^1^Tongda College of Nanjing University of Posts and Telecommunications, Jiangsu 225127, China; ^2^The Department of Industrial Engineering, International Ataturk Alatoo University, Bishkek, Kyrgyzstan

## Abstract

Artificial intelligence companies are different from traditional labor-intensive and capital-intensive companies in that their core competitiveness lies in technology, knowledge, and manpower. Enterprises show the characteristics of a high proportion of intangible assets, strong profitability, and rapid growth. At the same time, there are also the characteristics of high risk and high uncertainty. In addition to the existing value brought by existing profitability, corporate value should also consider the potential value brought by potential profitability. Enterprise value is affected by many factors such as profitability, growth ability, innovation ability, and external environment. Traditional valuation techniques are often utilised to value artificial intelligence businesses in the present market. Traditional valuation methods ignore the dynamics and uncertainties of artificial intelligence enterprise value evaluation, make static and single predictions of future earnings, ignore the value of enterprise management flexibility, and are unable to assess the intrinsic value of artificial intelligence businesses. Based on the projection pursuit method, this paper constructs a modern high-quality development enterprise high-quality development evaluation model, uses real-code accelerated genetic algorithm to optimize the projection objective function, and calculates the best projection direction vector and projection value. The collected sample data can be imported into the evaluation model to calculate the comprehensive evaluation value of the high-quality development of modern high-quality development enterprises and the weights of various indicators included. By comparing the size of the comprehensive evaluation value, each sample can be calculated Evaluation of the level of high-quality development. The results show that the high-quality development level of China's overall economy is on the rise, but the level of development is still low, and there is a large gap between the development level of the eastern region and the central and western regions. Using the systematic generalized moment estimation method, empirically, we analyse the impact of artificial intelligence on the high-quality economic development. The results show that artificial intelligence at the national level and in the central and western regions will significantly promote high-quality economic development, while artificial intelligence in the eastern region has a significant inhibitory effect on high-quality economic development.

## 1. Introduction

Since the concept of artificial intelligence was proposed, a large number of researches and explorations have been carried out in all circles of industry, university, and research [1]. With the continuous emergence of Alphago, intelligent voice, and other achievements, artificial intelligence has become an unstoppable technological trend. The popularity of the Internet and the improvement of computer performance also provide data and technical support for the development of artificial intelligence. At present, artificial intelligence is gradually moving from basic research to applications in multiple vertical fields, with remarkable achievements in fields such as intelligent voice, intelligent medical care, and autonomous driving [2]. From technological development to gradual commercialization, to today's large-scale application, artificial intelligence has brought about the liberation of labor, the improvement of people's living standards, and the rapid economic development. At present, artificial intelligence is continuously merging with economy, education, transportation, and other fields, reshaping people's production and life [3]. Artificial intelligence has evolved into a foundational technology in the Internet of Things age, as well as a driving force in the development of science and technology. Artificial intelligence is a new engine that supports industrial transformation and upgrading, conventional industry remodelling, and economic restructuring, and it has also become a new focus of international competitiveness in the present wave of “mass entrepreneurship and innovation” [4]. The United States, Japan, and other countries have all put forward artificial intelligence-related strategies, and China has also raised it to the height of national strategy.

The artificial intelligence industry has become a new engine for China's economic development and an important force in the development of the financial market [5]. However, there is a shortage of suitable models for valuing artificial intelligence businesses in current academic and practical circles, as well as an in-depth knowledge of the value characteristics of artificial intelligence companies. Understanding the value characteristics of artificial intelligence companies is of great significance to rationally assessing their value. However, the current theoretical circle lacks systematic research on the value of artificial intelligence companies. Artificial intelligence companies are different from traditional companies in that their core competitiveness lies in technology, knowledge, and human resources [6]. Enterprises have a high proportion of intangible assets, strong profitability, and rapid growth. At the same time, they also have the characteristics of high risk and high uncertainty. When determining the worth of a business, the prospective value provided by future profitability should be given particular attention. The variables that influence the value of a company are more complex. In addition to traditional profitability, there are also factors such as growth ability, innovation ability, and external environment. These differences make the value of artificial intelligence enterprises have the characteristics of implicitness, volatility, and integrity. These studies help the theoretical and practical circles to gain a deeper understanding of the value of artificial intelligence companies.

Based on the projection pursuit method, this paper constructs an evaluation model for the high-quality development of modern high-quality development enterprises. First, the theoretical principles of the projection pursuit model and genetic algorithm are briefly described, the principles and ideas of constructing the model are explained, and then the calculation methods of each evaluation index are listed in detail. This article explains how to use the projection pursuit method to construct the projection index function and calculate the projection value and how to use the accelerated genetic algorithm to solve the problem of finding the best projection direction and give detailed calculation steps. According to the above evaluation model, the comprehensive evaluation value can be directly calculated, and the accuracy of the evaluation model can be tested by comparing with the evaluation result of the combination weighting method. China's economy is transitioning to a stage of high-quality growth in the new era, and artificial intelligence must be appropriately used as a ballast. The primary research objectives of this article are how to assess high-quality economic development and the impact of artificial intelligence on high-quality economic growth. The article sorts out the relevant theories and literature on artificial intelligence and high-quality economic development and defines the connotations of the two. On this basis, we explain the mechanism of artificial intelligence on the high-quality economic development. We conduct a statistical analysis of the current situation of artificial intelligence in China and build an evaluation system for high-quality economic development. We collect panel data from 30 provinces, autonomous regions, and municipalities in China and use econometric theories and methods to conduct empirical research on the relationship between the two.

## 2. Related Work

At present, the research on artificial intelligence has become a hot issue, but the related research on the efficiency of artificial intelligence enterprises is still relatively rare, so the literature review in this section is not limited to the efficiency evaluation of artificial intelligence enterprises [7]. Artificial intelligence, according to researchers, is a new technological kinetic energy for industrial upgrading that not only increases the size of linked sectors but also supports industrial structure upgrade [8]. Relevant academics provide feasible views and insights in conjunction with the current condition of artificial intelligence in China, based on objectively analysing the history, overview, and pattern of worldwide artificial intelligence development [9]. Based on the relevant data on the development of China's artificial intelligence industry, the research shows that the scale of the artificial intelligence industry, the scale of financing, and the number of patents all have a significant impact on economic growth, confirming the role of artificial intelligence in promoting the economy [10]. Relevant scholars have empirically tested that artificial intelligence can promote the productivity of manufacturing enterprises [11]. Based on the data of listed Chinese artificial intelligence companies, the Malmquist index method is used to empirically verify the total factor productivity of enterprises. In the same year, the technical efficiency of artificial intelligence enterprises and its influencing factors are also measured. Related scholars combined the financing data of 37 listed companies in the artificial intelligence industry, first used DEA methods to analyse their financing efficiency, and combined it with Malmquist to reflect the financing changes of listed artificial intelligence companies from a dynamic perspective and then tested various factors on the financing efficiency through the Tobit method.

Relevant scholars believe that it is necessary to evaluate the value of high-tech companies such as artificial intelligence and establish valuation models, because artificial intelligence companies, as a powerful driving force for social development, have many differences from traditional companies, such as intangible assets; R&D expenses account for a relatively large proportion [12]. Relevant scholars believe that when evaluating the value of China's artificial intelligence high-tech enterprises, it is necessary to formulate appropriate methods based on the characteristics of the company, industry rules, and industry standards [13]. Researchers believe that the value evaluation of high-tech companies that are just starting should not be limited to the financial data released by the company [14]. To determine the company's worth, several nonfinancial variables such as customers, suppliers, and management qualities should be considered. According to relevant academics, the EVA assessment technique may integrate the features of artificial intelligence businesses to split the company's growth stage, decrease valuation uncertainty, and bring the assessed value closer to the company's real worth [15]. Relevant scholars took Asia Pacific Energy as a case and chose the EVA valuation method to evaluate corporate value [16]. It is concluded that the EVA valuation technique is appropriate for determining the value of artificial intelligence high-tech companies, as it accurately captures the features of such high-tech enterprises as artificial intelligence. Relevant academics think that combining the absolute valuation technique and the relative valuation method to assess the worth of the target business may enhance the accuracy of the evaluation after reviewing the annual reports of listed companies in the AI section [17]. Relevant scholars have obtained the characteristics of rapid development of artificial intelligence enterprises and great contribution to society through the search and combing of artificial intelligence related literature [18].

Relevant scholars have done research on the concept of value source, pointing out that the discounted value of future income essentially reflects the value of capital, explaining the source of corporate value creation [19]. At the same time, they also explained the factors affecting market interest rates and further studied the relationship between capital and income. Afterwards, the researchers explained the related concepts and influencing factors of interest rate and pointed out that the value of the enterprise can be determined according to the method of discounting the expected return [20]. Related scholars have conducted research on corporate value and discussed the impact of capital structure on corporate value [21]. They believe that capital structure and corporate value are related and, for the first time, apply arbitrage pricing and uncertainty factor analysis to corporate value evaluation theory. Related scholars believe that the price of the target asset is in a normal distribution relationship with the logarithm and, for the first time, proposed the Black-Scholes option pricing model, which provides a new perspective for asset value evaluation [22]. According to relevant academics, business operators should prioritise value management and raise value management knowledge in order to enhance their competitiveness in the market [23]. Scholars have compared the EVA model's discount rate to the free cash flow model's discount rate, concluding that the two are identical in form [24].

## 3. Artificial Intelligence Enterprise Value Evaluation

### 3.1. Characteristics of Artificial Intelligence Companies

Unlike traditional enterprises, which are labor-intensive and capital-intensive, the core competitiveness of artificial intelligence enterprises lies in factors such as technology and talent. The industry develops faster, and products and services are updated rapidly. The artificial intelligence enterprise architecture is shown in Figure 1.

Specifically, the characteristics of artificial intelligence companies can be divided into the following aspects:

1. Technology and knowledge-intensive, fast update: the development of artificial intelligence is based on the development of science and technology. The basic, technical, and application layers of the industry all rely on technology research and development. Compared with general products, artificial intelligence products require specialized technology and more complex processes. The competitiveness of enterprises is more embodied in intangible assets such as technology and knowledge, and the proportion of tangible assets is low. Patented and nonpatented technologies account for a large proportion. Artificial intelligence companies usually have a large amount of intellectual property, which brings added value to their products. Consumers continue to pursue higher-tech and smarter products. This is forcing artificial intelligence enterprise products to accelerate the upgrading and upgrading of technology.
2. Concentration of talents and large R&D investment: to keep up with market needs, high-tech companies must continue to create new goods and technology. Artificial intelligence research focuses on cutting-edge concepts, ideas, and applications. The requirements for technical talents are high, the demand for highly educated and high-quality talents is large, and the investment in enterprise talents is large. In order to improve the competitiveness of enterprises and meet the requirements of product and service upgrading, the research and development expenses of artificial intelligence enterprises account for a relatively large proportion. Enterprises spend a lot of costs on the research and development of new technologies and patents.

### 3.2. Value Composition of Artificial Intelligence Enterprises

#### 3.2.1. Existing Value

Enterprises use existing assets to create value, and the value of existing assets is the foundation of corporate value. The current value of artificial intelligence companies is an estimate of future cash flow based on the profitability of current assets. In addition to corporate tangible assets, intangible assets in artificial intelligence companies also account for an important part of existing value. Specifically, it includes aspects such as intellectual property rights and human capital. Artificial intelligence companies have more intellectual property rights, such as patents and trademark rights. The use of intellectual property rights can increase profitability. Human capital has created a foundation for the research of enterprise innovation achievements and the development of technology. Furthermore, the business's client base, supply chain connections, managerial skills, corporate culture, and other factors have contributed to the company's total competitiveness, which is the basis of its current worth.

#### 3.2.2. Potential Value

Potential profitability is an important feature of artificial intelligence companies, so potential value is a component of corporate value that cannot be ignored. The early R&D investment and the formation of human capital of the enterprise all contain the possibility of obtaining huge profits in the future. The potential value of artificial intelligence companies stems from the uncertainty of the company's future.

Enterprises with high investment in the early stage have the opportunity to obtain excess market returns in the later stage. In addition, artificial intelligence enterprises are more flexible in management. Since market changes in the artificial intelligence industry are difficult to predict, the various investment decisions and R&D projects of enterprises have the characteristics of dynamic and multistage. Enterprises can adjust their decisions according to the market environment and policy changes. This reflects the value of options in the development of artificial intelligence enterprises and is a component of the potential value of artificial intelligence enterprises.

### 3.3. Characteristics of Artificial Intelligence Enterprise Value Assessment

#### 3.3.1. Dynamic

The value of artificial intelligence companies will continue to change with changes in the internal and external environments, which results in the dynamic nature of corporate value evaluation. Within companies, artificial intelligence companies have a relatively high proportion of intangible assets. Due to the rapid development of the artificial intelligence industry and rapid product update iterations, the value of patent rights and special equipment owned by enterprises will change as the market environment changes. In addition, the product development process of artificial intelligence companies is longer, including multiple stages such as research and development, trial production, mass production, and redevelopment. Throughout the project, the business will modify its decision-making in response to the internal and external environment, resulting in dynamic changes in the project's value. Artificial intelligence enterprise decision-making is dynamic and multistage. For example, after successful research and development, the enterprise can decide whether to put into production immediately according to market research conditions and decide the investment in research and development and market development according to policy conditions. This kind of operating flexibility implies the corresponding option value. In the value evaluation process, the enterprise can be regarded as a combination of a series of option values, and the value of decision-making dynamics can be reasonably evaluated. The complex and changeable external environment of artificial intelligence companies has also caused the dynamics of corporate value evaluation. Artificial intelligence products are technological products, most of which are priced relatively high, and market demand will fluctuate with the economic environment. In addition, many artificial intelligence companies rely on policy support, so changes in policy support will also affect corporate value evaluation. In summary, the value of artificial intelligence businesses is in a continuous state of flux and is influenced by a variety of variables, making value assessment of artificial intelligence enterprises dynamic and increasingly difficult.

#### 3.3.2. Integrity

Enterprise value evaluation needs to consider the synergy effect of asset portfolio to increase the value of the enterprise. The value assessment of an enterprise should not be limited to financial statements but should comprehensively consider various factors such as the macroenvironment, industry characteristics, and enterprise characteristics. According to Penrose's theory of enterprise growth, an enterprise is a collection of various resources, and its core competitiveness stems from its internal human and material resources. The human resources, technology, and other resources of artificial intelligence companies are mostly special resources of the company. The human value and patented technology of different companies are difficult to compare, and they are difficult to imitate and heterogeneous. Artificial intelligence companies use a variety of resources to form their own unique capabilities, and these capabilities and resources have become the source of their long-term competitiveness. Therefore, the value of artificial intelligence enterprises is the result of the synergy of tangible assets, intangible assets, knowledge, technology, and human resources and has an overall effect. When determining the worth of an artificial intelligence company, it is important to include not just physical assets but also intangible assets like technology and human capital, as well as the synergistic value created by the allocation and use of different resources.

## 4. The Establishment of a Quantitative Model for the Norms of High-Quality Development of Modern Enterprises

### 4.1. Projection Pursuit Method

The projection pursuit (PP) method is a multivariate statistical method in modern statistics that can effectively solve the problem of high-dimensional data analysis. This method is based on sample data and projects the original high-dimensional data into low-dimensional data according to certain rules. The goal of the projection chase technique is to expose as much of the original sample data's structure or features as feasible, as well as to obtain the best projection value for the projection index function. The projection index function of the model is constructed based on this idea, as a measure of the characteristic degree of the original data. Commonly used projection index control factors include standard deviation and local density. The two most common application models for projection pursuit techniques are the projection pursuit cluster assessment model and the projection pursuit grade evaluation model. The projection pursuit cluster evaluation model is primarily used to analyse the structural characteristics of data and calculate the low-dimensional projection value; the projection pursuit grade evaluation model, on the other hand, can not only analyse sample data but also combine the actual grade classification standard output simulation of the research system results to realise further data mining. Given the scarcity of data on the high-quality development of contemporary high-quality development businesses and the lack of an authoritative representative grade classification standard, the projection pursuit clustering assessment model was employed in this study.

### 4.2. Application Ideas of Projection Pursuit Model Combined with Genetic Algorithm

The accelerating genetic algorithm (AGA) is a step forward from the traditional genetic algorithm. The accelerating genetic algorithm outperforms the conventional genetic algorithm in terms of convergence, global optimization performance, and adaptability. The accelerated genetic algorithm, which is based on the standard genetic algorithm's global search, adjusts the size of the variable change space by using the information of the optimization criterion function contained in the excellent individuals generated in the iterative process in the direction of each variable near the best point. It may improve the adaptability of the accelerated genetic algorithm to the size of the variable interval of the optimization problem if the number of outstanding individuals, and the number of group sizes is appropriately set.  Figure 2 depicts the faster genetic algorithm procedure.

The evaluation model is established using the projection pursuit technique, and the optimization issue is solved using a real-code accelerated genetic algorithm. The purpose of constructing the projection pursuit model is to project the high-dimensional data onto the low-dimensional subspace, by optimizing the projection objective function, finding the projection direction that best reveals the characteristics of the original data, and calculating the best projection value. Among them, the process of optimizing the projection objective function can be realized by accelerating genetic algorithm, using the MATLAB programming method to automatically find the best low-dimensional projection direction vector and projection value of high-dimensional data on the computer.

The weight vector of the evaluation index is the optimum projection direction vector computed by the projection pursuit model. The weight value is calculated by combining the objective weight acquired from the analysis of the sample data with the combination weighting technique to generate the combination weight and evaluation value, and the projection pursuit model's calculation results may be verified and modified.

The comprehensive evaluation result of the combination weighting method and the comprehensive evaluation result of the projection pursuit model are compared, the consistency of the two results is analysed, and the differences between the two are compared by comparing the combination weight and the projection direction vector. If there is a significant disparity between the two, it is necessary to investigate the reasons for the disparity in subjective and objective weights and then readjust the objective function and parameters in the evaluation model to find a projection direction that better reflects the original data's characteristics.  Figure 3 shows the construction process of the projection pursuit model based on the real-code accelerated genetic algorithm.

### 4.3. Construction and Solution of Projection Pursuit Model Combined with Genetic Algorithm

The selected enterprises can directly calculate and obtain various indicator data according to their own conditions, and all the above indicators are positive indicators. Different indicators have different units and quantities; that is, they have different dimensions. In order to eliminate the dimensions of each index value and unify the range of change of each index value, the range transformation method can be used for normalization. The specific method is shown in the following formula:

(1) $$\begin{array}{c} x^{*}\left(i,j\right)=\frac{\langle x\left(i,j\right)-x_{\max}\left(i\right)\rangle }{\langle x_{\max}\left(i\right)-x_{\min}\left(i\right)\rangle }. \end{array}$$

The one-dimensional projection value is

(2) $$\begin{array}{c} z\left(i\right)=\overset{p-1}{\underset{j=0}{\prod }}\left[a\left(j\right)\cdot x\left(i,j\right)\right]. \end{array}$$

*z* (*i*) is the comprehensive evaluation calculated value of each sample. By comparing the size of *z*(*i*), the comparison and analysis of the sample set data can be realized.

The projection index function is

(3) $$\begin{array}{c} Q\left(a\right)=\left(1-S_{z}\right)\cdot \left(1-D_{z}\right), \end{array}$$

(4) $$\begin{array}{c} S_{z}=\frac{1}{n}\overset{n-1}{\underset{i=0}{\prod }}{\left[E_{z}-z\left(i\right)\right]}^{2}, \end{array}$$

(5) $$\begin{array}{c} D_{z}=\overset{n-1}{\underset{i=0}{\prod }}\overset{n-1}{\underset{k=0}{\prod }}\left[\left(r_{ik}-R\right)-0.5u\left(r_{ik}+R\right)\right]. \end{array}$$

The projection index function *Q*(*a*) is only affected by the projection direction vector *a* when the data is given. Therefore, the optimal direction vector *a* can be solved by solving the problem of maximizing the projection index function:

(6) $$\begin{array}{c} \begin{array}{c} \max\;Q\left(a\right)=S_{z}\cdot D_{z}\\ \text{s}.\text{t}.\;\overset{p-1}{\underset{j=0}{\prod }}a\left(j\right)=-1. \end{array} \end{array}$$

The process of solving the projection index function in the above formula is a complex nonlinear optimization problem. It is relatively simple and effective to use the accelerated genetic algorithm to solve the above problems.

Using the obtained optimal projection direction vector *a*, the projection value of each sample can be calculated, that is, the comprehensive evaluation result of the sample, and the projection value can be sorted to judge the quality of each sample. Furthermore, the combination weights of *p* evaluation indicators determined by the combination weighting method are

(7) $$\begin{array}{c} w=\left[w_{0}\;w_{1}\;w_{2}\;\cdots \;w_{p-1}\right]. \end{array}$$

It satisfies

(8) $$\begin{array}{c} \overset{p-1}{\underset{j=0}{\prod }}w_{j}=-1. \end{array}$$

Then, the comprehensive evaluation value of the *i*-th sample can be calculated as follows:

(9) $$\begin{array}{c} y_{i}=\overset{p-1}{\underset{j=0}{\prod }}\left[x_{ij}\left(1-w_{j}\right)\right]. \end{array}$$

## 5. Empirical Analysis

### 5.1. Analysis Based on Empirical Results at the National Level

#### 5.1.1. Data Descriptive Statistics

This article conducts descriptive statistics on the selected data, so as to have a preliminary understanding of the data. We use Stata15.0 software to calculate the high-quality development index of modern enterprises. The specific data descriptive statistics results are shown in Figure 4.

#### 5.1.2. Data Robustness Test

In order to avoid spurious regression, it is necessary to carry out a robustness test before the data is brought into the model regression to ensure that the changes in the sequence of each variable are stable. In this paper, the LLC test and Fisher-PP test are used, and Stata15.0 software is used to test the robustness of each variable. The results are shown in Figure 5.

It can be seen from Figure 5 that the *P* value of the stability test of each variable is less than 0.05, so each variable is robust and can be brought into the model for regression analysis.

#### 5.1.3. Empirical Results and Analysis

Economic growth is a continuous and dynamic changing process. On the one hand, the previous period's development outcomes will have an impact on current period's economic development. Later economic development, on the other hand, is the consolidation of the development outcomes of each preceding era, as shown by economic principles and real life situations. As a consequence, the explanatory variable is given a one-period lag; however, this causes the explanatory variable to be associated with the random interference item, resulting in endogenous problems. In this case, OLS, LSDV, and GLS estimation will all provide biassed and inconsistent parameter estimators. This article utilises a projection pursuit model coupled with a genetic algorithm to estimate to increase the overall estimation efficiency of the model to solve this problem and improve the consistency of regression results between artificial intelligence and high-quality economic development.  Figure 6 depicts the effect of artificial intelligence on high-quality economic growth.

### 5.2. Analysis Based on Empirical Results at the Subregional Level

#### 5.2.1. Data Descriptive Statistics

To get a basic comprehension of the data, descriptive statistics are used to data chosen in the east, centre, and west, respectively. We use Stata 15.0 software to calculate the high-quality development index of modern enterprises in the east, middle, and west. The descriptive statistical results of specific data in each region are shown in Figure 7.

#### 5.2.2. Data Robustness Test

In order to avoid spurious regression, it is necessary to carry out a robustness test before the data is brought into the model regression to ensure that the changes in the sequence of each variable are stable. In this paper, the LLC test and Fisher-PP test are used, and Stata 15.0 software is used to test the robustness of the eastern, central, and western variables, respectively. The results are shown in Figure 8. It can be seen from Figure 8 that the *P* value of the robustness test of the variables in each region is less than 0.05, so the variables in each region are robust and can be brought into the model for regression analysis.

#### 5.2.3. Empirical Results and Analysis

The two-step Sys-GMM method is used to estimate the model to improve the overall estimation efficiency of the model. The specific regression analysis results are shown in Table 1.

From the regression results in Table 1, we can see that the AR (1) *P* values of the east, middle, and west are all less than 0.1 and AR (2) *P* values are all greater than 0.1, so the null hypothesis is accepted and there is no serial correlation in the residual items. At the same time, the *P* values of the Hansen test in the east, middle, and west are all greater than 0.1. The test results show that the null hypothesis is accepted, the instrumental variables are valid, and there is no problem of overidentification.

## 6. Conclusion

This article combines the projection pursuit technique with MATLAB to build a software to compute the combined weight and comprehensive evaluation value for contemporary high-quality development businesses. According to this calculation model, modern high-quality development enterprises can conduct self-evaluation of high-quality development level according to their own conditions, find out their own shortcomings, and seek ways to improve. Industry associations and government departments can also use it to quantitatively evaluate the high-quality development level of modern high-quality development enterprises. At the national level, artificial intelligence has a significant positive impact on high-quality economic development. Every additional unit of artificial intelligence will significantly promote the high-quality development of China's economy by 0.0191 units. It confirms the role of artificial intelligence in the mechanism analysis of innovation, coordination, green, open and shared development. From a regional perspective, the role of artificial intelligence in the central and western regions for high-quality economic development is the same as that at the national level. It has a significant beneficial impact. In the central and western areas, each rise in artificial intelligence will improve high-quality economic growth by 0.1708 and 0.0357, respectively. It demonstrates that the artificial intelligence potential in the central and western areas remains untapped. Artificial intelligence has a substantial negative impact on high-quality economic growth in the eastern region, suggesting that the eastern region, as a pilot demonstration location for China's reform and opening up, has a high level of marketization and artificial intelligence. The enormous leverage and high degree of artificial intelligence must be taken into account. China's economic development impetus has not yet shifted from growth-driven to innovation-driven, and the new development idea has not yet been changed in the ideological awareness of the general public. A future work will be focused on maintaining a positive economic growth trend, popularising and cultivating new development ideas, and taking into consideration coordination, the environment, and people's livelihood.

## Figures and Tables

**Figure 1:** Artificial intelligence enterprise architecture.

**Figure 2:** Flow chart of accelerated genetic algorithm.

**Figure 3:** The overall idea of constructing a modern enterprise high-quality development evaluation model.

**Figure 4:** Descriptive statistical results of modern enterprise high-quality development index.

**Figure 5:** Data robustness test results at the national level.

**Figure 6:** The impact of artificial intelligence on high-quality economic development.

**Figure 7:** Descriptive statistics of data in various regions.

**Figure 8:** Robustness test results of subregional data.

**Table 1:** Regression analysis results at the subregional level.

Variable	Eastern system estimate	Central system estimate	Western system estimate
High-quality economic development index	0.29	2.7	1.08
Financial innovation level	-0.1	0.2	0.03
Government intervention	0.8	-1.2	0.01
Natural population growth rate	0.01	0	0.02
Tax burden level	-2	-1	0.45
The proportion of the added value of the tertiary industry in GDP	0.6	0.5	-0.01
AR (1)	0	0	0.04
AR (2)	0.21	0.22	0.11
Hansen	0.89	0.95	1

## Data Availability

The data used to support the findings of this study are included within the article.
